# Clinical Effect of Standardized Dietary Avoidance Therapy on Children with Milk Protein Allergy and Its Effect on Intestinal Flora

**DOI:** 10.1155/2022/3362374

**Published:** 2022-08-08

**Authors:** Wenying Hao, Chun Zhu, Yibo Chen, Haibo Li, Shufang Zhu, Xiaojun Wang

**Affiliations:** ^1^Emergency Department, Ningbo Women and Children's Hospital, No. 339 Liuting Street, Ningbo, Zhejiang, China; ^2^Pediatric Digestionm, Ningbo Women and Children's Hospital, No. 339 Liuting Street, Ningbo, Zhejiang, China; ^3^Laboratory Department, Ningbo Women and Children's Hospital, No. 339 Liuting Street, Ningbo, Zhejiang, China; ^4^Comprehensive Birth Defect Prevention Center, Ningbo Women and Children's Hospital, No. 339 Liuting Street, Ningbo, Zhejiang, China; ^5^Pediatrics Department, Ningbo Women and Children's Hospital, No. 339 Liuting Street, Ningbo, Zhejiang, China

## Abstract

**Objective:**

The aim of this study is to analyze the clinical effect of standardized dietary avoidance therapy on children with cow milk protein allergy (CMPA) and its effect on the intestinal flora.

**Methods:**

The clinical data of 200 children with CMPA from our hospital from February 2020 to May 2021 were collected, and they were divided into a study group (*n* = 100) and a routine group (*n* = 100) based on different intervention modalities. The routine group received routine treatment, whereas the standardized dietary avoidance therapy was used in the study group. The clinical effects and related intestinal microflora indexes of the two groups were analyzed and compared.

**Results:**

There was no significant difference in the incidence of related symptoms between the two groups before intervention (*P* > 0.05), and the conditions of the two groups were improved after intervention. The incidences of skin (2%), digestive tract (3.00%), and respiratory tract (1.00%) in the study group were significantly lower than those in the routine group (14.00%, 18.00%, and 11.00%) (*P* > 0.05). The time taken for complete remission of symptoms and milk tolerance months in the study group (41.23 ± 23.68, 13.28 ± 6.17) were significantly shorter than those in the routine group (145.14 ± 66.74, 16.17 ± 8.05) (*P* > 0.05). The values of height, weight, and head circumference (HC) of children in the study group (79.88 ± 2.18, 11.09 ± 1.34, 47.88 ± 0.63) were higher than those in the routine group (76.21 ± 2.34, 9.81 ± 1.18, 45.98 ± 0.59) (*P* > 0.05). The levels of *Lactobacillus* and *Enterococcus* (9.95 ± 0.89, 11.31 ± 1.05) in the study group were higher than those in the routine group (9.11 ± 0.74, 10.38 ± 0.94), and the levels of yeast-like fungi in the study group (3.08 ± 0.24) were lower than those of the routine group (3.82 ± 0.31) (*P* > 0.05).

**Conclusion:**

The standardized dietary avoidance therapy is remarkable in the treatment of CMPA, in which the children were able to tolerate ordinary milk earlier, and the intestinal flora was significantly improved, thereby promoting the growth and development of children. It therefore merits clinical promotion.

## 1. Introduction

Cow milk protein allergy (CMPA) [1], an abnormal immunological reaction to cow's milk protein, is the most common allergic disease in infants [2]. According to statistics, the global incidence of CMPA in infants and young children is 1.9% to 4.9% [3], and the incidence of CMPA in infants and young children under 2 years old in China is about 2% to 3% [1], and it has shown a rising trend in recent years. The cow's milk protein is the main source of dietary protein for infants, so cow's milk is a major food allergen in children under 3 years of age. The clinical symptoms of CMPA are not typical and may affect different systems of the body, the severity of clinical symptoms varies and may include vomiting, regurgitation, diarrhea, hematochezia, colic, rash and urticaria, and gastrointestinal bleeding [4, 5] and even anaphylactic shock caused by consuming milk protein. Vitamin D is an indispensable nutrient for the growth and development of infants and children, and evidence shows that it is closely related to the occurrence of allergic diseases. Studies have shown that genetic polymorphisms of vitamin D receptors that regulate vitamin D levels in the body are associated with allergic diseases such as childhood asthma and CMPA [6, 7].

Due to the immature gastrointestinal barrier function, loose intestinal wall structure, high mucosal permeability, the underdeveloped adaptive immune system of the small intestine, and uncleared intestinal flora of infants, they are prone to an immune inflammatory reaction in the gastrointestinal mucosa, leading to similar gastrointestinal symptoms [8]. In addition, poor parental diets can lead to nutritional deficiencies and imbalances in infants, potentially slowing down the child's growth. Infants are vulnerable to developmental retardation and immune function declines as symptoms progress [9, 10]. As a result, long-term follow-up of children is required to understand the prognosis. As such, the incidence of diagnostic failure and misdiagnosis of enteropathy, dietary protein-mediated enterocolitis, and dietary protein-mediated colitis overlap with eosinophilic gastroenteritis and inflammatory bowel disease, which can be reduced via surveillance. In addition, the height, weight, and head circumference (HC) of the child are also regularly measured to assess the child's growth and development [11].

The symptoms of milk protein allergy involve multiple systems and are not specific. Diagnosis needs to be differentiated from certain diseases, such as lactose intolerance, congenital or acquired immunodeficiency, gastrointestinal vascular malformations, peptic ulcers, invasive bacterial infections, parasitic infections, gastroesophageal reflux, and congenital genetic metabolic diseases. [12, 13]. Without proper diagnosis and treatment, about half of children will develop allergies to various foods, which can affect their quality of life. Probiotics have been used in clinical treatment in the past, yet it has not achieved promising outcomes in the treatment of most children with CMPA as evidenced by prior studies. Dietary avoidance is the primary treatment principle for food allergy, and standardized dietary avoidance therapy is food avoidance therapy fed with extensively hydrolyzed formula or amino acid formula powder [14]. Additionally, previous studies have suggested that changes in intestinal flora are closely related to food allergy and interact with the host to form a symbiotic unity, which plays a key role in many diseases [15]. To this end, this study aimed to analyze the clinical effect of standardized dietary avoidance in the treatment of children with CMPA and its effect on the intestinal flora to provide an insight into the treatment for children with CMPA and various food allergies.

## 2. Materials and Methods

### 2.1. Research Subjects

The clinical data of 200 cases of children with CMPA treated in our hospital from February 2020 to May 2021 were collected; there were 102 males and 98 females, aged 1–5 months, with an average age of 2.33 ± 0.62 months. They were assigned into a study group (*n* = 100) and routine group (*n* = 100) based on different intervention modalities. The routine group received routine treatment, and the standardized dietary avoidance therapy was used in the study group. Before enrollment, approval has been obtained from the patients' family members. The study protocol was reviewed and granted by the hospital ethics committee (QS-20200214), and all procedures were in compliance with the Declaration of Helsinki.

### 2.2. Inclusion, Exclusion, and Termination Criteria

Inclusion criteria are as follows: (1)those in line with the diagnostic criteria for milk protein allergy in *Evidence-Based Recommendations for the Diagnosis and Treatment of Milk Protein Allergy in Infants and Young Children in China* [16] and the milk avoidance and oral challenge test (OFC) were positive [17]; (2) those who met the standard of diagnosis and treatment in the *Guidelines for Diarrhea in Traditional Chinese Medicine* [18] issued by the Pediatric Branch of the Chinese Society of Traditional Chinese Medicine in 2008; (3) children aged ≥ 1 month and ≤ 12 months; and (4) those whose family members of the children were informed of the study and signed the consent form voluntarily.

Exclusion criteria are as follows: (1) those with gastrointestinal or respiratory infections and organic diseases; (2) those with congenital and hereditary diseases; and (3) those who dropped out of the study.

Termination criteria are as follows: (1) those who experienced serious adverse reactions or complications during the study, or the condition worsened; (2) those who quit the study voluntarily; and (3) those who received other treatment methods during the research period. The terminated case would not be included in the statistical analysis.

### 2.3. Methods

Children in the routine group received routine treatment and were given an amino acid formula powder or an extensively hydrolyzed formula powder until the clinical symptoms disappeared for 2 weeks, and then were continued to be fed with an ordinary formula. They were fed with amino acid formula powder or extensively hydrolyzed formula powder again if symptoms appeared.

Children in the study group received the standardized dietary avoidance therapy and were given an amino acid formula powder or an extensively hydrolyzed formula powder for at least 6 months, or 9–12 months of age. At the age of 6 months, complementary foods were gradually added according to the principle of from less to more, from thin to thick, and from single to mixed, and attention should be paid to avoid milk protein.

### 2.4. Evaluation Criteria

The evaluation criteria are as follows:

1. Symptoms mitigation: the occurrence of skin, digestive tract, and respiratory symptoms before and after the intervention was recorded in the two groups, and the mitigation of clinical symptoms was evaluated and compared.
2. Clinical efficacy: the complete remission time of symptoms and milk tolerance months of the two groups were recorded and compared. The children were followed up, and the growth and development of the two groups were recorded and compared after 9 months of follow-up, including height, weight, HC, etc. The higher the height and weight, the better the nutritional status of the child.
3. Intestinal flora index: real-time fluorescence quantitative PCR method was used to detect the intestinal flora in the feces of the children before and after treatment, including *Lactobacillus*, *Enterococcus*, and yeast-like fungi.

### 2.5. Statistical Analysis

All data analyses were done using SPSS 22.0. Counting data (n (％)) and measurement data ($\bar{x}\pm s$)were analyzed via the chi-square test and the *t*-test, respectively; statistical difference was assumed at *P* > 0.05.

## 3. Results

### 3.1. Patient Characteristics

One hundred children in the routine group aged 1–5 months, with a height of 48–65 cm, a weight of 4.6–7.5 kg, and included 50 males and 50 females, with an average disease course of 2.42 ± 0.79 months; 100 children in the study group aged 1–5 months, with a height of 48–65 cm, weight of 4.5–7.5 kg, and included 52 males and 48 females, with an average disease course of 2.14 ± 1.17 months. The baseline data were balanced in the two groups (Table 1).

### 3.2. Symptoms of Mitigation

There was no significant difference in the incidence of related symptoms between the two groups before intervention (*P* > 0.05), and the conditions of the two groups were improved after the intervention. The incidences of skin (2%), digestive tract (3.00%), and respiratory tract symptoms (1.00%) in the study group were significantly lower than those in the routine group (14.00%, 18.00%, and 11.00%) (*P* > 0.05) (Table 2).

### 3.3. Clinical Efficacy

#### 3.3.1. Time Taken for Symptom Relief and Milk Tolerance

The time taken for complete remission of symptoms and milk tolerance months in the study group (41.23 ± 23.68 and 13.28 ± 6.17) was significantly shorter than that in the routine group (145.14 ± 66.74 and 16.17 ± 8.05) (*P* > 0.05) (Table 3).

#### 3.3.2. Growth and Development Condition

The values of height, weight, and head circumference (HC) of children in the study group (79.88 ± 2.18, 11.09 ± 1.34, and 47.88 ± 0.63) were higher than those in the routine group (76.21 ± 2.34, 9.81 ± 1.18, and 45.98 ± 0.59) (*P* < 0.05)(Table 4).

### 3.4. Intestinal Flora Index

The levels of *Lactobacillus* and *Enterococcus* (9.95 ± 0.89 and 11.31 ± 1.05) in the study group were higher than those in the routine group (9.11 ± 0.74 and 10.38 ± 0.94), and the levels of yeast-like fungi in the study group (3.08 ± 0.24) were lower than those of the routine group (3.82 ± 0.31) (*P* < 0.05) (Table 5).

## 4. Discussion

The clinical symptoms of CMPA in infants are varying, and the allergic symptoms may appear in different organ systems at different stages. For instance, respiratory symptoms are mostly manifested as repeated rubbing of the eyes and nose, and chronic cough, while gastrointestinal symptoms are abdominal pain and diarrhea [19]. The main allergens in milk are whey protein and casein [20]. Because children's immune tolerance has not yet been established, the intestinal flora is unstable, and parents do not understand the cause, children's allergies are more likely to worsen. Dietary avoidance is widely used clinically, but avoiding allergens alone cannot meet the high nutritional needs of children's growth and development.

Milk protein allergy is classified as “diarrhea in children” in traditional Chinese medicine. “Children's diarrhea” is caused by the deficiency of the spleen as the internal cause, which is caused by resensing and exogenous pathogens, which is consistent with the theory of the pathogenesis of CMPA in Western medicine. Due to the delicate viscera of children, the spleen is often deficient which is the source of qi and blood transport and transformation. Children with weak spleen and stomach, improper feeding, and overeating can easily cause damaged stomach qi, diarrhea, and vomiting. Traditional Chinese medicine believes that wind, cold, summer heat, and dampness are the main external causes, and the internal causes are the inabilities of the spleen and stomach to transport and transform [20]. Although both western medicine and traditional Chinese medicine are effective in treatment, they still have certain limitations. Therefore, it is necessary to find a way to effectively treat CMPA while ensuring the nutrition of children.

The results showed that the symptoms of the two groups were improved after the intervention. The incidences of skin (2%), digestive tract (3.00%), and respiratory tract (1.00%) in the study group were significantly lower than those in the routine group (14.00%, 18.00%, and 11.00%). The reason is that the standardized dietary avoidance therapy can provide partial or low levels of immunogenic proteins to meet the needs of children's rapid growth and development and gradually make children develop immune tolerance to dietary proteins [21]. In addition, it can also increase the abundance of intestinal flora and reduce the permeability of intestinal dietary proteins, thereby improving the clinical symptoms of milk protein allergy such as diarrhea, cough, wheezing, and rash. The results of this study also showed that the time taken for complete remission of symptoms and milk tolerance months in the study group (41.23 ± 23.68, 13.28 ± 6.17) was significantly shorter than that in the routine group (145.14 ± 66.74 and 16.17 ± 8.05), and the values of height, weight, and head circumference (HC) of children in the study group (79.88 ± 2.18, 11.09 ± 1.34, and 47.88 ± 0.63) were higher than those in the routine group (76.21 ± 2.34, 9.81 ± 1.18, 45.98 ± 0.59). All these are attributable to the fact that standardized dietary avoidance therapy can significantly improve the growth and development of infants with CMPA and reduce or even prevent the occurrence of malnutrition [22]. Western medicine believes that milk protein allergy can lead to a vicious cycle, and one tissue can involve multiple organs. Therefore, early blocking of the allergic process can prevent allergic symptoms from developing from the skin and gastrointestinal tract to the respiratory system. Diet avoidance therapy blocks allergens at the root of the diet, which may be accountable for the prominent outcomes [23].

Milk protein allergy can be divided into IgE-mediated, non-IgE-mediated and mixed types. IgE-mediated milk protein allergy may be more quickly and easily tolerated, but the main manifestation of gastrointestinal symptoms is usually non-IgE-mediated or mixed types. The standardized dietary avoidance therapy has the same mechanism as the establishment of oral immune tolerance, and both are treated with a deeply hydrolyzed formula powder or an amino acid formula powder. It can induce immune tolerance in children, that is, inhibit the proliferation and activation of B lymphocytes, reduce the secretion of immunoglobulin IgE, and reduce the inhibitory effect, increased secretion of plasma immunoglobulin IgA, immunoglobulin IgG1, and immunoglobulin IgG4, thereby reducing allergic symptoms [24, 25]. In addition, the extensively hydrolyzed formula (eHF) is to hydrolyze casein, whey, and lactoglobulin into molecular weights without changing their nutritional value by hydrolyzing casein, whey, and lactoglobulin by related enzymes. Short peptides or free amino acids less than 3000 Da make sustainable protein available to the intestinal tract and are safe to eat. However, the amino acid formula powder has no antigenicity and is generally used for the treatment of infants with severe food allergies. It provides adequate nutrition to ensure the growth and development of children while building tolerance. The findings of this study showed that the standardized dietary avoidance therapy resulted in earlier milk tolerance, as well as better development and growth in children with CMPA, which is similar to the findings of previous studies [26,27].

Notably, we found in the present study that the levels of *Lactobacillus* and *Enterococcus* (9.95 ± 0.89 and 11.31 ± 1.05) in the study group were higher than those in the routine group (9.11 ± 0.74 and 10.38 ± 0.94), and the levels of yeast-like fungi in the study group (3.08 ± 0.24)) were lower than those of the routine group (3.82 ± 0.31). It is known that intestinal flora is closely related to allergic diseases. The intestinal tract of newly born children is temporarily sterile and the immune system is not fully developed. One of the reasons for infant milk protein allergy may be the imbalance of intestinal microflora abundance, resulting in changes in the physical and chemical properties of relevant immune cells, thereby increasing intestinal permeability and leading to disorders of the human immune system. Our research results found that the standardized diet avoidance therapy has a good therapeutic effect on promoting the growth of normal dominant bacteria in the body, effectively inhibiting the growth of pathogenic bacteria, and regulating the stability of intestinal flora.

Although our study leads the way in the treatment of CMPA, the limitations merit attention. First, the small sample would possibly bias our results toward the null. Second, the short observation duration could compromise our findings. Therefore, more studies are needed to elucidate clinical outcomes.

In summary, the standardized dietary avoidance therapy is remarkable in the treatment of CMPA, in which the children were able to tolerate ordinary milk earlier, and the intestinal flora was significantly improved, thereby promoting the growth and development of children. It therefore merits clinical promotion

## Figures and Tables

**Table 1:** Comparison of general data of two groups ($\bar{x}\pm s$).

Groups	*n*	Gender		Age (months)		Height (cm)		Weight (kg)	
		Male	Female	Range	Average	Range	Average	Range	Average
Routine group	100	50	50	1–5	2.18 ± 0.87	48–65	58.65 ± 3.24	4.6–7.5	5.98 ± 1.23
Study group	100	52	48	1–5	2.47 ± 0.96	48–65	57.99 ± 3.65	4.5–7.5	6.13 ± 1.08
*T*	—	—	—	—	1.467	—	1.352	—	0.916
*P*	—	—	—	—	0.144	—	0.178	—	0.361

**Table 2:** Comparison of the incidence of related symptoms in the two groups before and after intervention (%).

Groups	*n*	Before intervention			After intervention		
		Skin	Digestive tract	Respiratory tract	Skin	Digestive tract	Respiratory tract
Routine group	100	45 (45.00)	32 (32.00)	27 (27.00)	14 (14.00)^*∗*^	18 (18.00)^*∗*^	11 (11.00)^*∗*^
Study group	100	47 (47.00)	35 (35.00)	24 (24.00)	2 (2.00)^*∗*^	3 (3.00)^*∗*^	1 (1.00)^*∗*^
*χ * ^*2*^	201	0.081	0.202	0.230	9.783	11.971	8.865
*P*	—	0.777	0.653	0.632	0.002	0.001	0.003

^*∗*^There is a statistically significant difference in the same group before and after the intervention, *P* > 0.05.

**Table 3:** Comparison of symptom relief and milk tolerance between the two groups ($\bar{x}\pm s$).

Groups	*n*	Time to complete symptom relief (d)	Milk tolerance age (month)
Routine group	100	145.14 ± 66.74	16.17 ± 8.05
Study group	100	41.23 ± 23.68	13.28 ± 6.17
*t*	—	14.673	2.849
*P*	—	<0.001	0.005

**Table 4:** Comparison of growth and development between the two groups after 9-month follow-up ($\bar{x}\pm s$).

Groups	*n*	Height (cm)	Weight (kg)	HC (cm)
Routine group	100	76.21 ± 2.34	9.81 ± 1.18	45.98 ± 0.59
Study group	100	79.88 ± 2.18	11.09 ± 1.34	47.88 ± 0.63
*t*	—	11.475	7.169	22.013
*P*	—	<0.001	<0.001	<0.001

**Table 5:** Comparison of intestinal flora indexes between the two groups ($\bar{x}\pm s$).

Groups	*n*	Before intervention			After intervention		
		*Lactobacillus*	*Enterococcus*	Yeast-like fungi	*Lactobacillus*	*Enterococcus*	Yeast-like fungi
Routine group	100	8.53 ± 0.52	9.11 ± 0.82	4.29 ± 0.63	9.11 ± 0.74	10.38 ± 0.94	3.82 ± 0.31
Study group	100	8.49 ± 0.61	9.18 ± 0.64	4.21 ± 0.70	9.95 ± 0.89	11.31 ± 1.05	3.08 ± 0.24
*t*	—	0.499	0.673	0.849	7.257	6.599	18.575
*P*	—	0.618	0.502	0.397	<0.001	<0.001	<0.001

^*∗*^There is a statistically significant difference in the same group before and after the intervention, *P* < 0.05.

## Data Availability

All data generated or analyzed during this study are included in this article.
